# Investigation on the Status Quo of Ecological Environment Construction in Northeast China from the Perspective of Dual Carbon Goals

**DOI:** 10.1155/2022/8360888

**Published:** 2022-09-19

**Authors:** Ailing Zhu

**Affiliations:** Changchun University, Changchun City, Jilin Province 130000, China

## Abstract

Since the 20th century, the resources and environment in Northeast China have changed, and it is one of the typical regions that have short-term or high-intensity environmental impacts in the world. However, due to the excessive consumption of regional resources and strong environmental pollution to the atmospheric environment, development is being greatly affected. Maintaining the natural ecological environment has become a very urgent task. This paper studies the important ecological environment problems in Northeast China from the perspective of double carbon goals. The study points out that there are ecological problems in Northeast China, such as the lack of forest resources, the aggravation of desertification, the decline of black soil quality, and the shrinkage of wetlands, which are severe urban environmental protection problems. At the same time, affected by the trend of world environmental change, policy drivers in Northeast China, and some relatively new environmental pollution problems, the natural environmental quality of Northeast China will still have a significant decline in the future. The future development of Northeast China will be based on the perspective of double carbon goals, constantly improve the ecological environment monitoring system, strengthen the research of scientific and technological system, strengthen innovation, and vigorously develop circular economy and further improve the construction of basic systems. Through a series of ecological environment governance and the coordinated development of economy and ecological environment, the dual growth of economy and ecological environment in Northeast China will be realized, and the overall revitalization of the old industrial zone in Northeast China will be realized.

## 1. Introduction

The northeast part is Liaoning, Jilin, and Heilongjiang, including three cities and one league in the east of Inner Mongolia (Chifeng City, Tongliao City, and Yilun City and Xing'an League). The overall framework of ecosystem is reasonable, especially suitable for the development of large-scale agriculture. It has been an important agricultural production base since ancient times and also an important industrial base in China [1]. According to the data at the end of 2014, the territorial area of the whole region is about 1.25 million square kilometers, which is 13% of the territorial area of the whole city; the population is about 118 million, accounting for 8.4% of the population of the province; the regional GDP is about 1.6 trillion, accounting for 11.8% [2]. Through the construction of nearly half a century, Northeast China has formed a large industrial system dominated by heavy industries such as steel, machinery, petroleum, chemical industry, and coal mining. It is China's main heavy industry production base and commodity grain production base and has a decisive strategic position for the development of Quantong. However, in the past two decades, the growth of enterprises in Northeast China has been slow, and their relative importance in China has decreased significantly. In addition to the problems of economic system, a series of ecological and environmental problems arising from the extensive development mode have restricted the development of Northeast China at the cost of natural resource consumption and environmental pollution damage for a long time.

The ecological environment is dominated by human settlements, including human survival and living environment, working environment, tourism environment, and resource cultivation environment [3]. Therefore, the ecological environment directly affects the life and quality of life of the creator of social productivity.

The natural environment is the basic condition for people's survival and development and is an important cornerstone of human economic and social development. Strengthening the construction of ecological environment, disaster prevention, and mitigation is an inevitable requirement for sustainable development.

Since the central government clearly puts forward a major strategic decision to revitalize the northeast and other old industrial training bases in 2003, environmental engineering has become one of the main focuses of scholars' research on revitalizing the Northeast [4]. Over the past two decades, investment in the construction of Northeast China has increased, and the development of the national economy has accelerated significantly. However, with the long-term historical accumulation, there are still many severe ecological and environmental problems, and the carrying capacity of resources and environment is also undergoing severe changes [5]. In order to further improve the existing natural ecological environment in Northeast China and realize the revitalization of the old industrial base, this paper systematically summarizes the main problems faced by the current ecological environment protection in Northeast China from the perspective of double carbon goals and predicts the recent development and changes of the ecological environment through possible influencing factors. Finally, the report points out the key measures to speed up the construction of ecological environment in Northeast China from the perspective of sustainable development.

## 2. Status Quo of Ecological Environment Development in Northeast China

### 2.1. Major Ecological and Environmental Problems in Northeast China

Over the past hundred years, large-scale mining has seriously polluted the natural environment in Northeast China and highlighted contradictions. Since the 20th century, with the short-term, high-intensity, and large-scale development of human society, the natural environment in Northeast China has also undergone great changes. In the first half of the 20th century, the Russian and Japanese colonists arrogantly seized iron ore, coal, and other resources, especially forest resources, which brought great damage to the economic resources and natural environment of Northeast China.  Figure 1 shows the administrative location of the Northeast region. Geographically, China has the greater Hinggan Mountains and Erguna River in the southwest; the lesser Hinggan Mountains and Heilongjiang and Wusuli rivers in the northeast; Jilin Changbai Mountain area, Tumen River, and Yalu River in the southeast; and Yilehu in the north. Lishan is connected to the northern part of the Greater and Lesser Xing'an Mountains, forming a unique natural geographical environment surrounded by five waters and surrounded by mountains on all sides.

Since the founding of new China, it has become the most strategic old industrial base in China. Large-scale industrial development and environmental pollution remediation are relatively backward, resulting in great energy consumption in Northeast China, and unreasonable development has seriously deteriorated the ecological environment (Figure 2). Some researchers even believe that the ecological environment in Northeast China is close to an irreversible critical state. Generally speaking, the ecological environment in Northeast China mainly faces the following problems [6].

Northeast China used to be the largest forest production base in China, but due to the long-term “heavy cutting and light cultivation” and “taking more than giving,” the forest region suffered a serious shortage of recoverable forest resources in the mid-1980s. According to statistics, as in the early stage of enclosure construction, the number of natural forests in Hilly and semimountainous areas in Northeast and Eastern China has declined rapidly. The area of natural forests in the South has decreased from 65 million hectares to 57.87 million hectares, and the water volume per hectare has also decreased from 172 cubic meters to 84 cubic meters [7]. Today, these natural primary forests have become secondary forests, with significantly reduced quality and serious deterioration of ecological functions. Taking Liaoning as an example, because of the uneven cutting and replenishment of resources in recent years, coupled with human deforestation, the area of natural forests in this region began to decline, and the primitive forests also basically disappeared; the proportion of natural protection forests is relatively small, accounting for only 22.9% of the national natural forest area; what is unreasonable is that the area of middle-aged and young forests accounts for 81.8% of the national natural forest area, and nearly mature forests, mature forests, and over mature forests only account for 18.2% of the total national natural forest area. The function of natural ecological construction has been seriously weakened. The importance of forest ecosystems is self-evident, such as forest vegetation that can intercept rainfall during the rainy season, maintaining most of the water on the leaf surface and in the leaf litter, soil, and living tissues, thus reducing surface runoff. In particular, forest litter can form a protective film on the surface of the soil layer, maintain the balance of the internal structure of the soil layer, and reduce the erosion of rainfall; it can increase soil roughness, filter, and intercept and reduce surface runoff; litter can increase the concentration of organic matter in land plants, thereby improving soil composition and fertility and increasing water holding capacity.

The greatest impact of human activities on the western part of the Northeast Plain of China was the agricultural development in the 1930s, especially the large-area cultivated land reclamation in the early 1980s, which further affected the grassland landscape and led to huge destruction of animals and plants. Soil desertification in the west of the Northeast Plain is mainly reflected in soil desertification and farmland salinization [8]. As shown in Figure 3, the desertification area of this area has reached 72280.6 square kilometers, accounting for 22.2% of the total land area of the country. From the 1950s to the late 1980s, the scale of desertification in the region increased sharply, with an average annual increase of about 1.5%-3.7%; since the 1990s, the scale of regional desertification has reversed, but in general, the scale growth of regional desertification has been greater than the reversal. At present, the salinized land in this region is 33850.8 square kilometers, accounting for 10.44% of the total land area, and is growing at an average annual rate of 1.4% to 2.5%, especially in Jilin Province. According to statistics, the area of water and soil erosion has reached 3.15 million hectares, accounting for about 16.5% of the land area of Jilin Province; the grassland area in the west is 1.36 million hectares, of which 472000 hectares are salinized, accounting for 36.7% of the total area of the country, and 158000 hectares are gravelized, accounting for 11.6% of the country.

Northeast black soil is mainly distributed in the middle of Songnen Plain, with a total area of about 11 million hectares, accounting for 8.9% of the total land area of Northeast China. However, in the past, nearly 0.5 century, due to excessive cultivated land, about two-thirds of the farmland in the whole black soil area has suffered serious soil erosion and low fertility [9].

Northeast China is the most important wetland area of the Yellow River in China, which is mainly distributed in Sanjiang plain, Songnen low plain, Xialiaohe plain and coastal areas, Hulunbuir grassland, great and small Xing'an Mountains, and Changbai Mountain Tourism Group Co., Ltd. Wetlands used to be the main natural barrier in Northeast China, but since the founding of the People's Republic of China, with the large-scale reclamation of cultivated land, the scale of wetlands has decreased significantly, coupled with the interference of engineering construction and human factors, and the natural landscape of wetlands has gradually disappeared and has been more and more seriously damaged [10].  Table 1 shows the land transfer matrix of Heilongjiang Province from 2010 to 2018. The ecological role of wetland parks in resisting floods; controlling rainfall runoff, flood storage, and drought resistance; controlling climate; preventing soil erosion; purifying the environment; and protecting biodiversity has been significantly weakened.

Most of the urban air pollution in Northeast China has the typical characteristics of urban coal-fired air pollution. In the heating period, the urban ambient air quality is obviously inferior to that in the nonheating period, and fine particles are also the primary pollutants that directly affect the urban indoor air quality. The content of particulate matter in winter heating period in Liaoning Province is 1.3~1.5 times that in the nonheating period; at the same time, the sand dust pollutants in spring are obvious, and the total suspended particulate matter content is 1.6 times that in winter and 1.9 times that in summer. However, the coal-fired pollutants in the urban atmospheric environment of Jilin Province have not been completely treated, and the air pollution load formed by coal-fired during the heating period accounts for more than 40% of the air pollution load [11].

### 2.2. Status Quo of Ecological Environment Governance in Northeast China

In recent years, leaders at all levels and government departments have begun to recognize the important role of the ecological environment and are paying more and more attention to the ecological environment and actively take measures to strengthen the construction of the ecological environment [12]. For example, Jilin Province proposed to establish an “ecological, environmental protection, and benefit-based economic framework” during the “Tenth Five-Year Plan” period, taking into account the construction of the ecological environment while considering leapfrog development. However, there are still many deficiencies in the governance of the deity environment, which are mainly manifested in the following aspects:

First, basic theoretical research is insufficient. The current environmental construction work has not yet been guided by a systematic theory, and most of them are in a state of blind construction or in a state of headache and foot pain. There is no theoretical basis for ecological environment construction in a certain area. For example, the proportion and layout of factories, institutions, schools, dwellings, and green spaces, as well as the environmental capacity of various landforms and organisms, have not yet been coordinated by a systematic theory.

Second, the ecological environment value assessment system has not yet been formed. It is impossible to make a correct quantitative evaluation of a built ecological environment, so it is impossible to evaluate the pros and cons of a pre-constructed environmental facility [13]. Often, the public is right, the mother is right, and the leadership is difficult to make decisions. For example, it is impossible to quantitatively compare the ecological environment value of “Dalian City's Big Lawn Green Space Construction Ideas,” “Jilin City's Jilin Street Reconstruction Project,” and so on.

Thirdly, in the means of ecological environment construction, the technological content is low, the technical level is not high, the construction efforts are small, and some development activities are still at the cost of environmental damage.

The government has insufficient respect for the laws of nature in decision-making, lacks sufficient demonstration, always follows others, and fails to get out of its own characteristics; human factors dominate the construction process, and the planning and design of some new communities are unreasonable. The green space rate is low, the awareness of advanced protection is lacking, and the strategic view of long-term sustainable development is not reflected.

### 2.3. The Trend of Ecological Environment Change in Northeast China

In the context of environmental changes at home and abroad, according to the analysis of the driving factors of economic development in Northeast China, it shows that the ecological environment situation in Northeast China has not been optimistic since the recent medium term [14], mainly in the following aspects.

First, the temperature increased significantly and the rainfall decreased slightly. The harm to the ecological environment is obvious. Northeast China is one of the sensitive regions of climate change [15]. In the past 100 years, the average temperature in Northeast China has shown a significant growth trend, especially in the past 20 years, showing an unprecedented significant warming momentum. As shown in Figure 4, although the annual average evaporation in Northeast China shows a significant upward trend, the annual average rainfall shows a slight decrease trend, which has decreased by nearly 20-30 mm since the beginning of the 20th century [16]. Before the mid-1960s, there was abundant rainfall in Northeast China. From the late 1960s to the early 1980s, Northeast China has always been in a dry period. From the mid-1980s to the mid-1990s, this was a wet era. Since the mid-1990s, Northeast China has always been in a dry period. The region will enter the next drought period. The rise of temperature and the decrease of precipitation have caused adverse effects on the ecological environment in Northeast China. In particular, it has caused an important impact on the drought situation in the northeast and central and western regions. Scientific research has confirmed that the reduction of rainfall is the main manifestation of drought in the central and western regions of Northeast China, resulting in the decline of the natural environment [17].

Second, there are also many debts caused by environmental pollution, which are difficult to control. The deterioration trend is obvious. For a long time, the development of industrial economy in Northeast China has always been at the expense of environmental protection, heavy industrial production, and light environmental protection. In order to achieve the national mandatory production goals, it has led to serious historical debt of ecological environment protection [18]. At the same time, as an old industrial base in Chinese history, heavy chemical industry has always accounted for a large proportion. Coupled with the development of coal and the energy pattern dominated by electricity, the ecological damage and pollution in Northeast China are coupled, making it more difficult to control [19].

Third, economic growth has accelerated, but structural transformation is difficult. The environmental pressure is further increased. Through the efforts of the whole 20th century, China's industrial system, which has the advantages of natural resource development and basic raw material resources, still has considerable advantages and will still play a key role in China's future economic development. According to their comparative advantages and economic foundation, the governments of the three northeastern provinces have focused on establishing a heavy industrial structure dominated by advanced equipment industry and raw material industry in their respective development plans. But it will still have a great burden on the earth's ecological environment [20]. Through several years of development, Northeast China will strengthen the modern industrial system dominated by heavy industries such as machinery and equipment industry, petrochemical industry, and metallurgy. Although the government has vigorously promoted the promotion of industrialization with informatization, actively promoted the development of high-tech manufacturing industry, and strengthened technological innovation, the system composed of heavy industry still determines that Northeast China will still be under greater environmental pressure in the future [21].

## 3. Analysis of the Causes of Ecological and Environmental Problems in Northeast China

### 3.1. The Traditional Development Model Induces the Occurrence of Ecological and Environmental Problems

The traditional mode of national economic development is a simple straight-line development of “natural resources, production, and environmental pollution utilization,” which is characterized by “high energy consumption, high emissions, low environmental volume, and low efficiency.” The sustainable basis of this approach lies in the inexhaustible, low-cost, and easy access of funds, and the preconditions on which this economic development model depends do not exist. Therefore, this development model is not sustainable for human society. The three northeastern provinces are China's old industrial bases and should adhere to the correct direction of sustainable development.

It is these traditional economic growth models that have been adopted for a long time at the expense of excessive consumption of natural resources and environmental protection. Although the three provinces have begun to actively explore and practice the new development path of circular economy, the traditional development model has induced and left over the utilization of resources. The contradiction between economic development and economic development, especially the grabbing and destruction of non-renewable productive resources, still has a negative impact on the ecological environment protection and development of this region.

### 3.2. The Level of Economic Development Restricts the Improvement of Ecological Environment

The emergence and worsening trend of ecological environment problems are inseparable from the long-term and frequent economic activities of human beings. From a practical point of view, the environmental problems of developed countries are gradually being solved and controlled, but the environmental problems of developing countries are generally not optimistic, which is closely related to the economic development level of developing countries.

The first is the influence of the traditional industrial development model. Industrialization is an insurmountable stage of development for any country. An important feature of the industrial structure of industrialization is that the heavy chemical industry occupies an important position in the development of the national economy. In terms of standard meaning, China's economy entered the primary stage of industrialization after the 1980s to meet the needs of the international market. At present, China's energy, transportation, metallurgy, chemical industry, building materials, and other heavily polluting industries are in a period of great development. Our economic development level is far from a stage where we can rely on scientific and technological progress to gradually improve the environment without affecting economic development. The mode of production of rural residents is relatively backward. Living standards are still generally low, and there is still a stage of over-grabbing of productive natural resources such as land and water, all of which put China's environment under heavy pressure and restrict the solution of environmental problems.

Secondly, the lack of environmental demand preference restricts the governance and improvement of the ecological environment. Increased government investment in environmental pollution control will inevitably affect investment in other economic activities. Therefore, in all developed countries, government departments cannot strengthen the ability of environmental pollution management without restrictions. This requires the government to make appropriate judgments and choices on environmental goals and the corresponding environmental pollution control efforts. Generally speaking, the choice of pollution control intensity is in line with people's environmental demand preference, and the strengthening of this demand preference is continuously improved with the improvement of economic level and education level. It cannot be arbitrarily strengthened by human will. From the perspective of the overall development level of China's economy, people's preference for environmental needs is not very strong, and this deficiency restricts the improvement of environmental problems to a certain extent. As a typical example of a planned economy, the three northeastern provinces have a large number of laid-off populations, and regional income levels are generally low. Coupled with factors such as culture, education, and technology, the characteristics of insufficient environmental demand preference are more obvious in the northeast. These are to a certain extent. It restricts the management and improvement of the ecological environment.

Third, the absence of the scientific concept of development artificially increases the emergence of ecological and environmental problems. If the first two factors are objective factors that are difficult to overcome in the short term, then the serious lack of the scientific development concept in the actual decision-making work is the main human factor that causes the current ecological and environmental problems and increases the environmental impact to a certain extent. Problem arises. For a long time, people lacked sufficient understanding of the importance of ecological construction and environmental protection in the process of sustainable economic and social development. The blind pursuit of GDP in economic life has led many departments to simply pursue the speed of economic development and is keen to do big projects and projects. In addition, due to the lack of scientific decision-making, some wrong decisions have been artificially expanded, further increasing the scope of environmental damage.

Finally, the defects of the public resource management system increase the difficulty of solving the ecological environment problem. One of the primary goals of transforming government functions is the realization of public management as the primary function of the government, which requires a series of institutional conditions to ensure its ability to regulate, as well as a series of institutional conditions to ensure that its behavioral goals conform to the interests of the people. However, at present, the government cannot guarantee the realization of these two conditions in the process of changing its functions, resulting in that many institutions that manage social public resources do not have sufficient institutional capacity. To some extent, it also improves the ability and difficulty of the government in dealing with ecological and environmental issues, as shown in Figure 5.

## 4. Significance and Countermeasures of Ecological Environment Construction in Northeast China

Although China's industrialization development stage is insurmountable, the traditional industrial development model can be changed, and the increasingly severe pressure on the ecological environment is destined to be urgent and necessary. The clear requirements of the new industrialization road on resource utilization and environmental protection provide a historic opportunity for the protection and improvement of the ecological environment in the three northeastern provinces.

### 4.1. Significance of Strengthening Ecological Environment Construction

One is the need for economic development. According to the data of some provinces, the direct loss caused by environmental damage in Northeast China is 100 billion yuan, indirect loss caused by ecological damage in Northeast China is about 10 million yuan, and the indirect economic loss, the restoration cost after ecological damage, and the potential economic loss that is difficult to measure in monetary terms are even greater. Only by strengthening the ecological environment protection and ensuring the environmental resource base for sustainable development can we realize the revitalization of the old industrial base in Northeast China and ensure the sustainable development of the economy in the Northeast region.

The second is the need for social development. Environmental pollution not only restricts the development of industrial and agricultural production but also destroys the living conditions on which people depend and endangers human health. Due to the deterioration of the ecological environment, the incidence of many diseases and fetal malformations in the industrial and mining areas are high. For example, the carcinogenic and teratogenic rates in Shenyang and Fushun areas were 1.2 times higher than those in the control areas. The increasing use of pesticides, chemical fertilizers, and agricultural film has led to the expansion of the polluted area of farmland and the decline of the quality of agricultural products. Northeast China is also China's commodity grain production base and the main heavy industry base. Improving and preserving the natural ecological environment in Northeast China are the basic requirements for the health of northeast people and the sustainable development of society, as well as the need for the national ecological environment protection.

### 4.2. Basic Ideas and Countermeasures for Improving the Ecological Environment in Northeast China

Compared with other regions of the country, the natural resources of Northeast China have their own unique advantages, but there are also some problems. In view of the problems existing in the utilization of environmental resources, governments at all levels and decision makers should provide a good sustainable development guarantee for the revitalization of the Northeast from the aspects of improving the system construction and promote the transformation and economic revitalization of the old industrial areas in the Northeast.

The first is to do a good job in the mechanism construction of ecological environmental protection. People's governments at all levels should give priority to environmental protection and incorporate the basic state policy of environmental protection into the macrostrategy of social and economic development. As shown in Figure 6, according to the ecosystem approach, rationalize the management system and build a multiagent comprehensive governance model. Promote the improvement of laws and regulations, improve the scientific decision-making and supervision mechanism, improve the supervision system, and create a good legal and regulatory environment for the implementation of effective macro-control. Establish and improve the responsibility system of people's governments at all levels for the quality management of the ecological environment under their jurisdiction and of all units for the management of industrial and social environment. Improve the ecological environmental protection and management audit system, and implement a strict performance reward and punishment system. Establish and improve the subsidy system for natural resources and environmental protection, and increase the investment in natural resource protection and development. Establish and implement tax relief measures, tax relief measures, credit preferential policies, and other relevant measures to ensure that the ecological environment work in Northeast China is carried out well.

The second is to adjust the industrial structure and change the mode of economic growth. Industry in Northeast China, especially heavy industry, has an absolute advantage in the economy, and the industrial structure is unreasonable. At the same time, most cities belong to resource-based heavy industry cities, and the environmental pollution is relatively serious. Although environmental protection and pollution control have been intensified and environmental quality has improved, the overall environmental situation has not been fundamentally improved. Transform the mode of economic development, promote the development of industrial technological transformation, vigorously implement the policy of industrial energy conservation and consumption reduction, and form an economic mode of energy conservation, and promote the coordinated development of the urbanization process and the ecological environment. While the regional urban space reconstruction has an impact on the ecological environment, it is also responded by the ecological environment. The feedback itself can hinder or accelerate the process of urban space reconstruction and affect the effect of urban space reconstruction as shown in Figure 7.

Thirdly, actively participate in environmental protection cooperation in Northeast Asia. Northeast Asia is the region with the largest number of neighbors and the most extensive contacts in Northeast Asia, and it is also an ideal region for international cooperation in Northeast Asia. The development of environmental cooperation among countries in Northeast Asia is an external condition necessary for the development of Northeast old industrial bases. Regional environmental cooperation in Northeast Asia can promote the environmental governance and environmental quality improvement of key river basins, regions, and cities in Northeast China. For example, Heilongjiang Province used yen loans to support the prevention and control of water pollution in the Songhua River Basin. Through the regional environmental cooperation in Northeast Asia, international advanced environmental concepts and environmental management experience are introduced to improve the level of environmental protection technology, governance technology, and other environmental technology cooperation. These have a good reference and enlightenment for revitalizing the northeast old industrial base.

## 5. Conclusion

Ecological environment is an eternal topic that the majority of residents, especially the government management and decision-making departments, urgently need to pay attention to. It is related to people's health and living standards. Ensuring and improving the basic conditions for people's survival and promoting sustainable development are the fundamental strategies for China's economic growth. Under the guidance of the new concept of development, the formation of a new mode of growth plays a major role in the overall development of the regional ecological environment and economic and social development. China is rapidly industrializing. “WTO entry” has accelerated her pace of integration into economic globalization. The launch of the “Northeast Revitalization Project” has opened an important scene of northeast industrial structure adjustment. In the new era, the economic development of the three northeastern provinces is facing new major opportunities. Ecological construction and environmental protection are also facing new challenges. The phenomenon of ecological environment in Northeast China is particularly obvious, which has caused harm to the sustainable development of local social economy and the revitalization of the old industrial base in Northeast China. The northeast ecological construction and environmental protection strategy in the new era are of far-reaching significance for promoting the revitalization of old industrial bases and sustainable economic and social development. On the basis of objective research and scientific understanding of the major natural resource ecological and environmental problems that need to be solved urgently in this region, we should actively take positive measures to improve the legal system, increase scientific and technological investment, and promote the adjustment of industrial structure, so as to do a good job in ecological construction, use ecological energy scientifically, promote the ecological environment, and promote regional development and sustainable economic and social development.

## Figures and Tables

**Figure 1:** Schematic diagram of the geographical location of Northeast China.

**Figure 2:** Ecological and environmental problems in Northeast China.

**Figure 3:** Map of desertification in the western part of the Northeast Plain of China.

**Figure 4:** Variation curves of annual average evaporation1 and precipitation2 in Northeast China.

**Figure 5:** Lack of local government public resource management system.

**Figure 6:** Ecoenvironmental governance in a multiagent model.

**Figure 7:** The synergistic mechanism of urbanization and ecological environment governance.

**Table 1:** Land transfer matrix of Heilongjiang Province from 2010 to 2018.

Area (km^2^) 2010	2018						
	Cultivated land	Woodland	Grassland	Waters	Land used for building	Unused land	Total
Cultivated land	159413.21	1084.84	584.80	161.28	980.91	636.74	162871.79
Woodland	2369.42	188756.58	431.27	57.32	78.58	2879.57	194572.74
Grassland	4696.25	1432.60	20191.65	280.92	136.80	8881.62	35619.85
Waters	2417.84	95.49	67.04	9226.58	65.53	1680.63	13553.11
Land used for building	313.80	16.89	14.65	25.33	9275.15	24.77	9670.60
Unused land	5627.41	467.61	718.06	410.38	116.28	28819.86	36159.60
Total	174837.93	191854.01	22017.47	10161.82	10653.26	42923.18	452447.68

## Data Availability

The labeled data set used to support the findings of this study is available from the corresponding author upon request.
